This article has been retracted.

# A Family of Optimal Multiple-Weight Optical Orthogonal Codes for Fiber-Optic Networks

**DOI:** 10.1155/2022/2499606

**Published:** 2022-05-23

**Authors:** Dandan Xu, Haitao Cao

**Affiliations:** ^1^Institute of Mathematics, Nanjing Normal University, Nan Jing 210023, China; ^2^Department of General Education, Army Engineering University of PLA, Nan Jing 211101, China

## Abstract

Optical orthogonal codes (OOCs) were designed for multimedia optical CDMA systems with quality of service requirements in optical fiber networks. Two-dimensional (2-D) multiple-weight optical orthogonal codes have been invested as they can overcome the drawbacks of nonlinear effects in large spreading sequences. In this paper, we reveal the combinatorial properties of optimal 2-D OOCs and focus our attention on the constructions for a family of optimal 2-D multiple-weight optical orthogonal codes by combinatorial methods, such as incomplete difference matrix, h-perfect cyclic packing, and skew starter. In particular, an improved construction of skew starters with multiple weights is also proposed to solve the existence of optimal multiple-weight optical orthogonal codes. Our numerical examples demonstrate that the proposed construction is very helpful for optimizing the utilization of optical network effectively.

## 1. Introduction

There has been a current application to deal with the requirement of high-speed access and local area networks through the growing techniques of optical networks. Optical code-division multiple access (OCDMA shortly) networks are attractive for their ability to support asynchronous, concurrent, and secure communications; in addition, their good performance in the presence of simultaneous multiple users in shared media increase the transmission capacity of the fiber-optic telecommunications. In fiber-optic CDMA networks, optical orthogonal codes (OOCs) are introduced. A one-dimensional constant-weight optical orthogonal code (1-D OOC) is a family of sequences with good auto-correlation and cross-correlation properties, which has acquired wide attention as signature patterns in an optical code-division multiple access system. For more details, the reader may refer to [1, 2] for more backgrounds on 1-D OOCs, and for recent results on 1-D OOCs.

As in the case of fiber optic communications, the drawback of 1-D OOCs is that the auto-correlation cannot be zero because there are more than one pulse within one period, and to implement auto-correlation; the code length increases as the number of users increases. In order to overcome this drawback, 2-D constant-weight OOCs were put forward. Currently, many researchers are interested in constructions and designs of 2-D constant-weight OOCs, see [3] for examples. However, a 2-D constant-weight OOC has an extremely restriction, which only can support a single quality service requirement. In [4], 2-D multiple -weight OOCs were introduced to meet multiple quality service requirements. A 2-D multiple -weight OOC has multiple Hamming weights. When a 2-D multiple-weight OOC is employed for encoding quality service for a distinct service can be supported. In doing so, the demands of different quality service for different services and distinct subscribers can be fulfilled and the utilization of optical network can be optimized. It seems that 2-D multiple-weight OOCs have the tremendous potential to be wide-ranging used. Hence, we will accomplish a new family of optimal 2-D (*n* × *m*, {3,4}, 1, {1/3, 2/3})-OOCs.

Throughout this paper, we suppose that *W*={*w*_1_, *w*_2_,…, *w*_*l*_} is an ordered set of *l* positive integers greater than one, Γ_*a*_={*λ*_*a*_^(1)^, *λ*_*a*_^(2)^,…, *λ*_*a*_^(*l*)^} a *l*-tuple of positive integers, *λ*_*c*_ a positive integers, and *Q*={*q*_1_, *q*_2_,…, *q*_*l*_} a *l*-tuple of positive rational numbers. A two dimensional-(*n* × *m*, *W*, Γ_*a*_, *λ*_*c*_, *Q*) multiple-weight optical orthogonal code, or briefly 2-D (*n* × *m*, *W*, Γ_*a*_, *λ*_*c*_, *Q*)-OOC, *ℂ*, is a family of *n* × *m* (0,1)-arrays with the multiple Hamming weight set *W* such that the following correlation properties hold:

(1) Weight distribution: Each codeword in *ℂ* has a corresponding Hamming weight contained in the set W; furthermore, *q*_*p*_ shows the fraction of code words of weight *w*_*p*_, 1 ≤ *p* ≤ *l*;
(2) Auto-correlation property: For any matrix *B*=(*b*_*ij*_) ∈ *ℂ* (0 ≤ *i* ≤ *n* − 1, 0 ≤ *j* ≤ *m* − 1) and any integers *δ* with 0 < *δ* < *m*,
  (1) $$\begin{array}{c} \overset{n-1}{\underset{i=0}{\sum }}\overset{m-1}{\underset{j=0}{\sum }}b_{ij}b_{ij{⊕}_{m}\delta }\leq \lambda_{a}^{\left(p\right)},\;1\leq p\leq l. \end{array}$$
(3) Cross-correlation property: For any two distinct matrices *D*=(*d*_*ij*_) ∈ *ℂ* (0 ≤ *i* ≤ *n* − 1, 0 ≤ *j* ≤ *m* − 1) and any integer *δ* with 0 < *δ* < *m*, where the addition ⊕_*m*_ is reduced modulo *m*,
  (2) $$\begin{array}{c} \overset{n-1}{\underset{i=0}{\sum }}\overset{m-1}{\underset{j=0}{\sum }}b_{ij}d_{ij{⊕}_{m}\delta }\leq \lambda_{c}. \end{array}$$

From the definition, it is straightforward to see that a 2-D (*n* × *m*, *W*, Γ_*a*_, *λ*_*c*_, *Q*)-OOC is nothing else but a one-dimensional (*n* × *m*, *W*, Γ_*a*_, *λ*_*c*_, *Q*) multiple-weight optical orthogonal code, or briefly 1-D (*v*, *W*, Γ_*a*_, *λ*_*c*_, *Q*)-OOC when *n*=1 and *m*=*v*. *As* to a 1-D (*v*, *k*, *λ*, 1)-OOC (constant-weight OOC) one means a 1-D (*v*, *W*, Γ_*a*_, *λ*_*c*_, *Q*)-OOC with *λ*_*a*_^(1)^=*λ*_*a*_^(2)^=⋯=*λ*_*a*_^(*l*)^=*λ*_*c*_=*λ*, *W*={*k*} and *Q*={1}. We can say that a multiple-weight optical orthogonal code (multiple-weight OOC) is a generalization of a constant-weight optical orthogonal code OOC (constant-weight OOC). The set *Q* is called normalized if it is considered as the form {*d*_1_/*c*, *d*_2_/*c*,…, *d*_*l*_/*c*}, where *c*, *d*_*i*_ are integers such that gcd(*c*, *d*_*i*_)=1, and gcd(*d*_1_, *d*_2_,…, *d*_*l*_)=1 , 1 ≤ *i* ≤ *l*. The number of codewords in a 2-D (*n* × *m*, *W*, Γ_*a*_, *λ*_*c*_, *Q*)-OOC is the size of the OOC and it is maximal when every other OOC with the same parameters has not greater than the number. For given values *n*, *m*, *w*_*i*_, *λ*_*a*_^(*i*)^, *λ* and *q*_*i*_, let Θ(*n* × *m*, *W*, Γ_*a*_, *λ*, *Q*) denote the maximal possible size of *co*  *de*  *wor*  *ds* among all 2-D (*n* × *m*, *W*, Γ_*a*_, *λ*, *Q*)-OOCs. Therefore, a 2-D (*n* × *m*, *W*, Γ_*a*_, *λ*, *Q*)-OOC will be said optimal when Θ(*n* × *m*, *W*, Γ_*a*_, *λ*, *Q*) reaches the upper bound in [1], which is stated below:

(3) $$\begin{array}{c} \Theta \left(n\times m,W,\Gamma_{a},\lambda ,Q\right)\leq \left\lfloor \frac{\left(nm-1\right)\left(nm-2\right)\cdots \left(nm-\lambda \right)}{\sum_{i=1}^{l}q_{i}w_{i}\left(w_{i}-1\right)\left(w_{i}-2\right)\cdots \left(w_{i}-\lambda \right)/\lambda_{a}^{\left(i\right)}}\right\rfloor . \end{array}$$

If *Q* is normalized and *λ*_*a*_^(1)^=*λ*_*a*_^(2)^=⋯=*λ*_*a*_^(*l*)^=*λ*_*c*_=1, we also can write the value Θ(*n* × *m*, *W*, 1, *Q*) as the following:

(4) $$\begin{array}{c} \Theta \left(n\times m,W,1,Q\right)\leq c\left[\frac{nm-1}{\sum_{i=1}^{l}d_{i}w_{i}\left(w_{i}-1\right)}\right]. \end{array}$$

Specially, when *W*={3,4}, *λ*=1 and *Q*={1/3, 2/3}, we get the upper bound for the fixed value of Θ(*n* × *m*, {3,4}, 1, {1/3, 2/3}) from (4). Speaking of an optimal 2-D (*n* × *m*, {3,4}, 1, {1/3, 2/3})-OOC, it is easy to show that the value Θ(*n* × *m*, {3,4}, 1, {1/3, 2/3}) reaches the upper bound of 3⌊*nm* − 1/30⌋.

We present some known results on optimal multiple-weight OOCs as the following. For the case *W*={3,4}, when *Q*={1/3, 2/3}, *n*=15, *m*=*u* and *u* ≡ 1(mod2), the existence of a 2-D(*n* × *m*, *W*, 1, *Q*)-OOC has been already solved in [5]; when *Q*={2/3, 1/3}, and *n* = 12, *m* = *u* or *n* = 1, *m* = 24*t* + 1 is a prime, there exists a 2-D(*n* × *m*,*W*, 1, *Q*)-OOC by [5]; for the case *Q*={1/2, 1/2}, see [6]. For some details on the constructions of optimal multiple-weight OOCs with *W*={{3,5}, {4,5}}, see [4]. One can refer to [2, 7] for weight 3, [6, 8, 9] for existing results on OOCs with weight 4, and [4] for OOCs with weight 5. For more results on multiple-weight OOCs with three or more different weights, the readers can refer to [5, 6, 10].

In this paper, we put our focus on the constructions of a new family of optimal 2-D (*n* × *m*, {3,4}, 1, {1/3, 2/3})-OOCs by using incomplete difference matrix, *h*-perfect cyclic packing, and skew starters, when *n* and *m* are not coprime.

## 2. Fundamentals

Optimal OOCs can be constructed from some combinational designs. The result in [1] has proved that a 1-D optimal (*m*, *k*, 1)-OOC is equivalent to an optimal cyclic difference packing. Similarly, optimal (*m*, *W*, 1, *Q*)-OOCs were constructed by the optimal cyclic difference packing given in [8]. Now, we first give some necessary definitions before giving our recursive constructions.

Suppose that *K* is a set of positive integers, a cyclic difference packing (namely, 2-CDP (*K*, 1; *m*)), is a difference family Λ={*D*_1_, *D*_2_,…, *D*_*l*_} of *l*-subsets (called base blocks) of *Z*_*v*_. Let Λ be the set {|*D*_*i*_| : 1 ≤ *i* ≤ *l*}={*k*_1_, *k*_2_,…, *k*_*s*_}, such that the differences in Λ, ΔΛ={*d*_*ij*_ − *d*_*is*_ : 1 ≤ *i* ≤ *l*,  1 ≤ *j* ≠ *s* ≤ |*D*_*i*_|}, cover each element in *Z*_*m*_\{0} at most once. A 2-CDP (*K*, 1; *m*) can be considered as a CDP (*K*, 1; *m*) in [4]. A CDP (*W*, 1, *Q*; *m*) is defined to be a CDP (*W*, 1; *m*) with the property that the fraction of number of base blocks of size *W*_*j*_ is *q*_*j*_, 1 ≤ *j* ≤ *s*, where *W*={3,4} and *Q*={1/3, 2/3}.

Assume that Λ is a CDP (*W*, 1, *Q*; *m*), for every *D* ∈ Λ , the list of differences from *D* is recorded as Δ  *D*={*c* − *d* : *c*, *d* ∈ *D*, *c* ≠ *d*}. Define ΔΛ=∪_*D*∈Λ_Δ  *D*. The difference leave of Λ, shortly DL(Λ), is the set of all nonzero positive integers in *Z*_*m*_ which are not covered by ΔΛ. A CDP (*W*, 1, *Q*; *m*) is g-regular if the difference leave DL(Λ) along with zero forms an additive subgroups of *Z*_*m*_ with its order *g*, which must be generated by integers *m*/*g*. The reader may refer to [6, 10] for more details.

The stated results are presented in [3].

**Lemma 1 .**

An optimal CDP (*W*, 1, *Q*; *m*) is equivalent to an optimal 1-D (*m*, *W*, 1, *Q*)-OOC.

**Lemma 2 .**

Let *Q*=(*d*_1_/*c*, *d*_2_/*c*,…, *d*_*l*_/*c*), and *t*=∑_*i*=1_^*l*^*d*_*i*_*t*_*i*_(*t*_*i*_ − 1). If 1 ≤ *g* ≤ *t*,   then a *g*-regular CDP (*W*, 1, *Q*; *m*) is optimal. Moreover, if there exists a *g*-regular CDP (*W*, 1, *Q*; *m*), then *m* ≡ *g*(mod*t*).

By Lemma 2, in order to construct optimal-OOCs, we need to describe its corresponding optimal CDP ({3,4}, 1, {1/3, 2/3}; *m*)*s*. From the abovementioned Lemmas, it is clear to get that the largest possible size of base blocks of a CDP ({3,4}, 1, {1/3, 2/3}; *m*) is 3⌊*m* − 1/30⌋. A CDP ({3,4}, 1, {1/3, 2/3}; *m*) is optimal if the value of its base blocks reaches this upper bound.

**Construction 1 .**

([10]) Suppose that both a *g*-regular CDP (*W*, 1, *Q*; *m*) and an optimal CDP (*W*, 1, *Q*; *g*) exist, then an optimal CDP (*W*, 1, *Q*; *m*) exists. Moreover, if the given CDP (*W*, 1, *Q*; *g*) is *r*-regular, then so is the desired CDP (*W*, 1, *Q*, *m*).

Difference array plays an important part in the recursive constructions of cyclic designs. Now, we give the definition of an incomplete difference matrix. Let (*G*, ·) be a finite group of order *m* and *H* a subgroup of order *h* in *G*. An *h*-regular (*m*, *kλ*)-incomplete difference array in *G* is a *k* × *λ*(*m* − *h*) matrix *C*=(*c*_*ij*_), 0 ≤ *i* ≤ *k*, 1 ≤ *j* ≤ *λ*(*m* − *h*), with entries from *G*, such that for any 0 ≤ *i* ≤ *j* ≤ *k* − 1, the set

(5) $$\begin{array}{c} \left\{c_{il}\cdot c_{jl}^{-1}:1\leq l\leq \lambda \left(m-h\right)\right\}. \end{array}$$

contains every element of*G*\*H* exactly *λ* times. When *G* is an abelian group, typically additive notation is used, so that (*c*_*il*_ − *c*_*jl*_) are employed. In what follows, we assume that *H* is a subgroup of order *h* in *Z*_*m*_. Here, let *H* =  {*i* · *m*/*h* : 0 ≤ *i* ≤ *h* − 1}.An*H*-regular (*m*, *k*; *λ*)-incomplete difference matrix over *Z*_*m*_ is usually denoted by *h*-regular (*m*, *k*; *λ*)-ICDM if |*H*|=*h*.An *H*-regular (*m*, *kλ*)-incomplete difference matrix over *Z*_*m*_ is termed as (*m*, *k*; *λ*)-CDM when |*H*|=Φ or *h* = 0.

**Lemma 3 ([6]).**

If *v* ≥ *k* is an odd prime, then there exists an (*v*, *k*; 1)-CDM.

**Lemma 4 ([6]).**

If *v* ≥ 5 is oddgcd(*v*, 27) ≠ 9, then there exists an (v, 4; 1)-CDM.

**Lemma 5 ([6]).**

There exists a 2-regular (*m*, 4; 1)-ICDM for *m* ∈ {12,18}, or *m*=2^*n*^ and *n* ≥ 3.

**Construction 2 .**

([6]) Suppose that there exist a g-regular CDP (*W*, 1, *Q*; *m*), an (*v*, *w*_*i*_; 1)-CDM, and an optimal CDP (*W*, 1, *Q*; *gm*). Then there exists an optimal CDP (*W*, 1, *Q*; *gm*). Moreover, if the given CDP (*W*, 1, *Q*; *gm*) is *r*-regular, then so is the derived CDP (*W*, 1, *Q*, *mv*).

For more constructions, we still need the definition of an h-perfect cyclic packing. Let *g* be a divisor of *v* such that *m* = *gm*_0_. Assume that Λ={*D*_*i*_,  *i*=1,2,…, *l*} is the family of base blocks of an hg-regular CDP (*W*, 1, *Q*; *hv*), where *D*_*i*_={0, *d*_1*i*_, *d*_2*i*_,…, *d*_*w*_*k*−1_,*i*_} for *w*_*k*_ ∈ *W*,  *k* ∈ {1,2,…, *r*}, and *i*=1,2,…, *l*. Define

(6) $$\begin{array}{c} ele\left(\Lambda \right)=\overset{l}{\underset{i=1}{\cup }}\left\{d_{1i},d_{2i},\ldots ,d_{w_{k-1},i}\right\}. \end{array}$$

The hg-regular CDP (*W*, 1, *Q*; *hv*) is said to be *h*-perfect, denoted by *hg*-regular *h*-perfect CDP (*W*, 1, *Q*; *hv*) when

(7) $$\begin{array}{c} ele\left(\Lambda \right)\subseteq \left\{c+dm\;:0\leq c\leq \left\lfloor \frac{m}{2}\right\rfloor ,\;c\neq 0,\;m_{0},2m_{0},\ldots ,\left(g-1\right)m_{0};\;d=0,1,2\ldots ,h-1\right\}. \end{array}$$

As the constructions presented in [5], the following two results are obtained.

**Construction 3 .**

Let *v* and *m* be positive integers such that gcd(*m*, *v*)=1.Suppose that there exist a g-regular CDP (*W*, 1, *Q*; *v*), an h-regular (*m*, *w*_*i*_; 1)-ICDM, and an *hg*-regular CDP (*W*, 1, *Q*; *hv*) (or a *gh*-regular CDP (*W*, 1, *Q*; *gm*), respectively). Then, there exists *angm*-regular CDP (*W*, 1, *Q*; *mv*) (or an *hv*-regular CDP (*W*, 1, *Q*; *mv*), respectively).

**Construction 4 .**

Let *v* and *m* be positive integers. Suppose that there exist a *g*regular 1-perfect CDP (*W*, 1, *Q*; *v*), an *hg*-regular *h*-perfect CDP (*W*, 1, *Q*; *hv*), and an *h*-regular (*m*, *w*_*i*_; 1)-ICDM. Then, there exists an mg-regular m-perfect CDP (*W*, 1, *Q*; *mv*).

## 3. Constructions Using Skew Starters

In this part, the definition of skew starters is first introduced, and some directed constructions for regular CDPs are given by using skew starters. Suppose (*G*; +) be an Abelian group of order *n* > 1. A skew starter in *G* is a set of unordered pairs

(8) $$\begin{array}{c} S=\left\{\left\{u_{i},v_{i}\right\}:1\leq i\leq \frac{\left(n-1\right)}{2}\right\}. \end{array}$$

which satisfies the following three properties:

1. {*u*_*i*_ : 1 ≤ *i* ≤ (*n* − 1)/2} ∪ {*v*_*i*_ : 1 ≤ *i* ≤ (*n* − 1)/2}=*G*\{0};
2. {±(*u*_*i*_ − *v*_*i*_) : 1 ≤ *i* ≤ (*n* − 1)/2}=*G*\{0};
3. {±(*u*_*i*_+*v*_*i*_) : 1 ≤ *i* ≤ (*n* − 1)/2}=*G*\{0}.

According to the abovementioned statement, a skew starter in *G* can exist only if *n* is odd. Let *U*={*u*_*i*_ : 1 ≤ *i* ≤ (*n* − 1)/2}, *V*={*v*_*i*_ : 1 ≤ *i* ≤ (*n* − 1)/2}, then, we may assume that *U*=−*V* and hence, we have *U* ∪ (−*V*)=*U* ∪ (−*V*)=*U* ∪ *V*=*G*\{0}. Skew starters have been used to construct constant-weight optical orthogonal codes and optimal multiple-weight OOCs. Then, following results are stated in [9].

**Lemma 6 .**

([5]) There exists a skew starter in *Z*_*m*_ for each positive integer *m* such that gcd(*m*, 150)=1 or 25. There does not exist any skew starter in *Z*_*m*_ if *m* ≡ 0 (mod 3).

According Lemma 6, we can obtain a skew starter in *Z*_*v*_, if gcd(*v*, 30) ≡ 1. In what follows, suppose that *ℜ* is a set of subsets *of* *Z*_*v*_ × *Z*_*g*_, define the list of differences

(9) $$\begin{array}{c} D_{s}=\left\{d:\left(d,s\right)\;is\;a\;di\;fference\;from\;ℜ\right\}. \end{array}$$

**Lemma 7 .**

Let *u* be a positive integer such that gcd(*v*, 150)=1 or 25, then there exists a g-regular CDP ({3,4}, 1, *Q*; *gu*) for (*Q*, *g*) ∈ {({1/3, 2/3}, 60), ({1/3, 2/3}, 90)}.

**Proof**

By applying Lemma 6, there exists a skew starter *S*={{*u*_*i*_, *v*_*i*_} : 1 ≤ *i* ≤ (*n* − 1)/2} in *Z*_*n*_. For gcd(*n*, 60)=1, *Z*_*n*_ × *Z*_*g*_ is isomorphic to *Z*_60*n*_. Then 6(n-1) base blocks of a 60-regular CDP ({3,4}, 1, {1/3, 2/3}; 60*n*) on *Z*_*n*_ × *Z*_60_ are listed as follows, where 1 ≤ *i* ≤ (*n* − 1)/2.

(10) $$\begin{array}{c} A_{i}^{1}=\left\{\left(u_{i},0\right),\left(v_{i},0\right),\left(u_{i}+v_{i},1\right),\left(0,31\right)\right\},\\ A_{i}^{2}=\left\{\left(u_{i},0\right),\left(-v_{i},7\right),\left(-u_{i},16\right),\left(v_{i},39\right)\right\},\\ A_{i}^{3}=\left\{\left(-u_{i},0\right),\left(v_{i},7\right),\left(u_{i},16\right),\left(-v_{i},39\right)\right\},\\ A_{i}^{4}=\left\{\left(u_{i},0\right),\left(-v_{i},3\right),\left(-u_{i},5\right),\left(v_{i},43\right)\right\},\\ A_{i}^{5}=\left\{\left(-u_{i},0\right),\left(v_{i},3\right),\left(u_{i},5\right),\left(-v_{i},43\right)\right\},\\ A_{i}^{6}=\left\{\left(u_{i},0\right),\left(-v_{i},8\right),\left(-u_{i},26\right),\left(v_{i},41\right)\right\},\\ A_{i}^{7}=\left\{\left(-u_{i},0\right),\left(v_{i},8\right),\left(u_{i},26\right),\left(-v_{i},41\right)\right\},\\ A_{i}^{8}=\left\{\left(u_{i},0\right),\left(v_{i},11\right),\left(-u_{i},36\right),\left(v_{i},47\right)\right\},\\ A_{i}^{9}=\left\{\left(0,0\right),\left(2u_{i}+2v_{i},12\right),\left(u_{i}+v_{i},25\right)\right\},\\ A_{i}^{10}=\left\{\left(0,0\right),\left(-2u_{i},6\right),\left(-2u_{i}-2v_{i},12\right)\right\},\\ A_{i}^{11}=\left\{\left(-u_{i},0\right),\left(v_{i},4\right),\left(u_{i},14\right)\right\},\\ A_{i}^{12}=\left\{\left(u_{i},0\right),\left(-v_{i},4\right),\left(-v_{i},14\right)\right\}. \end{array}$$

Now, we begin to calculate the difference from them. Since *D*_*s*_=−*D*_60−*s*_ *for* 30 ≤ *s* ≤ 59, we only need to consider *D*_*j*_ for 0 ≤ *j* ≤ 30. It is to be noted that gcd(*n*, 60)=1, set Λ={*A*_*i*_^*j*^ : 1 ≤ *i* ≤ (*n* − 1)/2, 1 ≤ *j* ≤ (*n* − 1)/2}. Then, ΔΛ covers each element of *Z*_*n*_ × *Z*_60_\({0} × *Z*_60_) exactly once, while any element of the additive subgroup {0} × *Z*_60_ is not covered at all. Hence, Λ forms a 60-regular CDP ({3,4}, 1, {1/3, 2/3}; 60*n*). Table 1 describes the differences of 60*n*, where *t*=(*n* − 1)/2.

The proof for (*Q*, *g*) = ({1/3; 2/3}, 90) is similar to that of (*Q*, *g*)=({1/3, 2/3}, 60), the base blocks of an optimal CDP ({3,4}, 1, {1/3, 2/3}; 90*n*):

(11) $$\begin{array}{c} A_{i}^{1}=\left\{\left(u_{i},0\right),\left(v_{i},0\right),\left(u_{i}+v_{i},1\right),\left(0,46\right)\right\},\\ A_{i}^{2}=\left\{\left(u_{i},0\right),\left(-v_{i},8\right),\left(-u_{i},37\right),\left(v_{i},76\right)\right\},\\ A_{i}^{3}=\left\{\left(-u_{i},0\right),\left(v_{i},8\right),\left(u_{i},37\right),\left(-v_{i},76\right)\right\},\\ A_{i}^{4}=\left\{\left(u_{i},0\right),\left(-v_{i},15\right),\left(-u_{i},43\right),\left(v_{i},64\right)\right\},\\ A_{i}^{5}=\left\{\left(-u_{i},0\right),\left(v_{i},15\right),\left(u_{i},43\right),\left(-v_{i},64\right)\right\},\\ A_{i}^{6}=\left\{\left(u_{i},0\right),\left(-v_{i},16\right),\left(-u_{i},48\right),\left(v_{i},72\right)\right\},\\ A_{i}^{7}=\left\{\left(-u_{i},0\right),\left(v_{i},16\right),\left(u_{i},48\right),\left(-v_{i},72\right)\right\},\\ A_{i}^{8}=\left\{\left(u_{i},0\right),\left(-v_{i},4\right),\left(-u_{i},67\right),\left(v_{i},77\right)\right\},\\ A_{i}^{9}=\left\{\left(-u_{i},0\right),\left(v_{i},4\right),\left(u_{i},67\right),\left(-v_{i},77\right)\right\},\\ A_{i}^{10}=\left\{\left(u_{i},0\right),\left(-v_{i},3\right),\left(-u_{i},5\right),\left(v_{i},38\right)\right\},\\ A_{i}^{11}=\left\{\left(u_{i},0\right),\left(v_{i},11\right),\left(-u_{i},20\right),\left(-v_{i},31\right)\right\},\\ A_{i}^{12}=\left\{\left(-u_{i},0\right),\left(v_{i},3\right),\left(u_{i},5\right),\left(v_{i},38\right)\right\},\\ A_{i}^{13}=\left\{\left(-u_{i},0\right),\left(v_{i},6\right),\left(u_{i},36\right.\right\},\\ A_{i}^{14}=\left\{\left(u_{i},0\right),\left(-v_{i},6\right),\left(-u_{i},36\right)\right\},\\ A_{i}^{15}=\left\{\left(-u_{i},0\right),\left(v_{i},7\right),u_{i},19\right\},\\ A_{i}^{16}=\left\{\left(u_{i},0\right),\left(-v_{i},7\right),\left(-u_{i},19\right)\right\},\\ A_{i}^{17}=\left\{\left(0,0\right),\left(2u_{i}+2v_{i},50\right),\left(u_{i}+v_{i},81\right)\right\},\\ A_{i}^{18}=\left\{\left(0,0\right),\left(-2u_{i},25\right),\left(-2u_{i}-2v_{i},50\right)\right\}. \end{array}$$

We begin to calculate the difference from them. Since *D*_*s*_=−*D*_90−*s*_ for 45 ≤ *s* ≤ 89, we need to consider *D*_*j*_ for 0 ≤ *j* ≤ 45. It is to be noted that gcd(*n*, 90)=1, *t*=(*n* − 1)/2, set Λ={*A*_*i*_^*j*^ : 1 ≤ *i* ≤ (*n* − 1)/2,  1 ≤ *j* ≠ (*n* − 1)/2}. Then, ΔΛ covers each element of *Z*_*n*_ × *Z*_90_\({0} × *Z*_90_) exactly once, while any element of the additive subgroup {0} × *Z*_90_ is not covered at all. So, Λ forms a 90-regular CDP ({3,4}, 1, {1/3, 2/3}; 90*n*). Then, Table 2 lists the differences of 90*n*.

In order to exhibit an improved method to get hg-regular CDP({3,4},1,*Q*; *gn*)s based on Lemma 6, we need the cyclic packing satisfied some special properties. It is clear that displayed below is very helpful to our discussions.

**Definition 1 .**

A(*W*,1,*Q*; *g*)-CDP, *F*, is called good, denoted by (*W*,1,*Q*; *g*)-GCP, if DL(*F*)={0, *g*/2, ±1, ±*g* − 2/2, ±*a*, ±*b*, ±(*a*+*b*), ±(*b* − *a*), ±2*b*, ±*g* − 2*b*/2} with |DL(*F*)|=18 when *g* is even, or DL(F) =  {0, ±*a*, ±2*a*, ±(*a*+1), ±(3*a*+1)} with |DL(*F*)|=9 when *g* is odd.

Starting from the GCPs, we can give the following construction of more g-regular CDP(*W*, 1, *Q*; *gn*)s.

**Construction 5 .**

Suppose a (*W*,1,*Q*; *g*)-GCP exists, where *W* = {3, 4}. Let *q*_0_ and *q*_1_ be the number of blocks of size 3 and 4, and *q*=*q*_0_+*q*_1_ . There exists a *g*-regular CDP (*W*, 1, {*q*_0_+1/*q*+2, *q*_1_+1/*q*+2}; *gu*) when *g* is even, or a g-regular CDP (*W*, 1,{*q*_0_+1/2*q*+2, *q*_1_+1/2*q*+2}; *gn*) when *g* is odd, for *n* is a positive integer such that gcd(*n*, 150) = 1 or 25.

**Proof**

By Lemma 6, there exists a skew starter *S*={{*u*_*i*_, *v*_*i*_} : 1 ≤ *i* ≤ (*u* − 1)/2} in *Z*_*n*_. Since gcd(*n*, *g*) = 1, *Z*_*n*_ × *Z*_*g*_ is isomorphic to *Z*_*gn*_. Suppose that *B* = {*B*_*j*_: *j* = 1, 2,…, *q*} is the family of base blocks of a (*W*, 1, *Q*; *g*)-GCP, where *B*_*j*_ = {0, *b*_1*j*_, *b*_2*j*_ ,…, *b*_*w*_*k*−1_,*j*_} for *w*_*k*_ ∈ {3,4}, *k* ∈ {1,2,3,4}, and *j* = 1, 2,…, *q*. If *B*_*j*_ = {0, *b*_1*j*_, *b*_2*j*_,…, *b*_*w*_*k*−1_,*j*_} ∈*B* for wk = 3, *B*_*j*_ is denoted as *B*_*j*_^1^={(*x*_*i*_, 0), (−*x*_*i*_, *b*_1*j*_), (*y*_*i*_, *b*_2*j*_)} and *B*_*j*_^2^  =  {(−*x*_*i*_, 0), (*x*_*i*_, *b*_1*j*_), (−*y*_*i*_, *b*_2*j*_)}, respectively, where 1 ≤ *j* ≤ *q*_0_ , 1 ≤ *i* ≤ (*u* − 1)/2 . If *B*_*j*_ = {0, *b*_1*j*_, b2j ,…, *b*_*w*_*k*−1_,*j*_ }∈*B* for *w*_*k*_ = 4, we denote *B*_*j*_ as *B*_*j*_^1^={(*x*_*i*_, 0), (−*y*_*i*_, *b*_1*j*_), (−*x*_*i*_, *b*_2*j*_), (*y*_*i*_, *b*_3*j*_)} and *B*_*j*_^2^  = {(−*x*_*i*_, 0), (*y*_*i*_, *b*_1*j*_), (*x*_*i*_, *b*_2*j*_), (−*y*_*i*_, *b*_3*j*_)}, respectively, where 1 ≤ *j* ≤ *q*_1_,  1 ≤ *i* ≤ (*n* − 1)/2. Considering the DL(F), it can be divided into two cases as following. For the case of *g* is even:

(12) $$\begin{array}{c} A_{1}=\left\{\left(x_{i},0\right),\left(y_{i},0\right),\left(x_{i}+y_{i},1\right),\left(0,\frac{g+2}{2}\right)\right\},\\ A_{2}=\left\{\left(x_{i},0\right),\left(y_{i},a\right),\left(-x_{i},b\right),\left(-y_{i},a+b\right)\right\},\\ A_{3}=\left\{\left(0,0\right),\left(-2x_{i}-2y_{i},-2b\right),\left(-x_{i},b\right),\left(-x_{i}-y_{i},a-b\right)\right\},\\ A_{4}=\left\{\left(0,0\right),\left(2x_{i},\frac{\left(g-2b\right)}{2}\right),\left(2x_{i}+2y_{i},-2b\right)\right\}. \end{array}$$

For the case of *g* is odd:

(13) $$\begin{array}{c} A_{1}=\left\{\left(x_{i},0\right),\left(y_{i},0\right),\left(x_{i}+y_{i},1+a\right),\left(0,3a+1\right)\right\},\\ A_{2}=\left\{\left(0,0\right),\left(x_{i},a\right),\left(x_{i}+y_{i},2a\right)\right\}. \end{array}$$

Now, we begin to calculate the difference from them. When *g* is even, since *D*_*s*_=−*D*_*g*−*s*_ *for* *g*+2/2 ≤ *s* ≤ *g* − 1, we need to consider *D*_*j*_ for 0 ≤ *s* ≤ *g*/2. Because of the diﬀerences of second coordinates from B appear in pairs, so the diﬀerences of corresponding ﬁrst coordinates satisfy the properties of the skew starter. If the diﬀerences of second coordinates from DL(F), then the proof details are listed in the following for brevity, where *t*=*n* − 1/2.

(14) $$\begin{array}{c} D_{1}=\overset{t}{\underset{i=1}{\cup }}\left\{\left(x_{i}+y_{i}\right)\right\},\\ D_{0}=\overset{t}{\underset{i=1}{\cup }}\left\{\pm \left(x_{i}-y_{i}\right)\right\},\\ D_{g-2b/2}=\overset{t}{\underset{i=1}{\cup }}\left\{\left(2x_{i},2y_{i}\right)\right\},\\ D_{-2b}=\overset{t}{\underset{i=1}{\cup }}\left\{\pm 2\left(x_{i}-y_{i}\right)\right\},\\ D_{g-2/2}=\overset{t}{\underset{i=1}{\cup }}\left\{\left(-x_{i},-y_{i}\right)\right\},\\ D_{b-a}=D_{b+a}=D_{g/2}=\overset{t}{\underset{i=1}{\cup }}\left\{\pm \left(x_{i}+y_{i}\right)\right\}. \end{array}$$

Similar to above, the case *g* odd can be obtained. Set *F*={*A*_*i*_ : 1 ≤ *i* ≤ 4} ∪ {*B*_*j*_^*m*^ : 1 ≤ *j* ≤ *q*, 1 ≤ *m* ≤ 2}. It is easy to check that △*F* covers each element of *Z*_*u*_ × *Z*_*g*_\({0} × *Z*_*g*_) exactly once, while any element of the additive subgroup {0} × *Z*_*g*_ is not covered at all. We also can computer the numbers of block size 3 and size 4 of *F* are 2*q*_0_+2 and 2*q*_1_+2 when *g* is even, respectively. The numbers of block size 3 and size 4 of *r* are 2*q*_0_+1 and 2*q*_1_+1 when *g* is odd, respectively. So, *F* forms the *g*-regular CDP(*W*, 1, *Q*; *gn*), where *Q*={*q*_0_+1/*q*+2, *q*_1_+1/*q*+2} when *g* is even, or *Q* =  {2*q*_0_+1/2*q*+2, 2*q*_1_+1/2*q*+2} when *g* is odd.

**Example 1 .**

If *u* > 1 is an integer such that gcd(*n*, 150) = 1, or 25, then there exists a *g*-regular CDP ({3, 4}, 1, *Q*; *gn*) for (*Q*, *g*) ∈ {({3/4, 1/4}, 45), ({7/8, 1/8}, 81), ({2/3, 1/3}, 48), ({2/5, 3/5}, 48), ({1/2, 1/2}, 54), ({3/4, 1/4}, 60), ({4/5, 1/5}, 72), ({1/3, 2/3}, 90)}.

**Proof**

By Construction 5, the required GCPs are listed in for details.

**Theorem 1 .**

Suppose that a *g*-regular CDP (*W*, 1, *Q*; *gu*) exists, where *W*={*w*_0_, *w*_1_,…, *w*_*p*_}. Let *q*_*l*_ be the number of blocks of size *w*_*l*_,  0 ≤ *l* ≤ *p*, and *q*=*q*_0_+*q*_1_+⋯+*q*_*p*_. If there exists a (W, 1, *Q*′; *g*)-GCP, where *q*_1_′ be the number of blocks of size *w*_*l*_,  0 ≤ *l* ≤ *p* and *q*′=*q*_0_′+*q*_1_′+⋯+*q*_*p*_′. then there exists a (W, 1, *Q*^″^; *gu*)-GCP for *Q*^″^={*q*_0_+*q*_0_′/*q*+*q*′, *q*_1_+*q*_1_′/*q*+*q*′,…, *q*_*p*_+*q*_*p*_′/*q*+*q*′}.

**Proof**

Suppose that *F*_1_={*C*_*i*_={0, *c*_1*i*_, *c*_2*i*_,…, *c*_*w*_*k*−1,*i*__} : *i*=1,2,…, *q*}, *w*_*k*_ ∈ *W* is a g-regular CDP (W, 1, *Q*; *gn*). Let *B*={*B*_*s*_={0, *b*_1*s*_, *b*_2*s*_,…, *b*_*w*_*k*−1,*s*__} : *s*=1,2,…, *q*}, *w*_*k*_ ∈ *W* be a g-regular GCP (*W*, 1, *Q*; g). Let *F*_2_={*uB*_*s*_={0, *ub*_1*s*_, *ub*_2*s*_,…, *ub*_*w*_*k*−1,*s*__} : *s*=1,2,…, *q*′}, where *ub*_1*s*_, *ub*_2*s*_,…, *ub*_*w*_*k*−1_,*l*_ ∈ {0, *u*,…, (*g* − 1)*u*}. Here, DL(F2) ⊆{*ua* : 0 ≤ *ua* ≤ *u*(*g* − 1)}. Consider the family:

(15) $$\begin{array}{c} \left\{\begin{array}{c} F_{1}=\left\{C_{i}=\left\{0,c_{1i},c_{2i},\ldots ,c_{w_{k-1,i}}\right\}:i=1,2,\ldots ,q\right\};\\ F_{2}=\left\{uB_{s}=\left\{0,ub_{1s},ub_{2s},\ldots ,ub_{w_{k-1,s}}\right\}:s=1,2,\ldots ,q\prime \right\},\\ \text{DL}\left(F_{2}\right)\subseteq \left\{ua:0\leq ua\leq u\left(g-1\right)\right\}. \end{array}\right. \end{array}$$

Now, set the family *F*=*F*_1_ ∪ *F*_2_.. It is clear that the sum of blocks of size *w*_*l*_ of F is *q*_*l*_+*q*_*l*_′,  0 ≤ *l* ≤ *p*. Since *F* is a (*W,* 1, *Q*^″^; *gu*)-GCP, where *DL*(*F*)⊆{*d*=*ua* : 0 ≤ *d* ≤ *u*(*g* − 1)} and *Q*^″^={*q*_0_+*q*_0_′/*q*+*q*′, *q*_1_+*q*_1_′/*q*+*q*′,…, *q*_*p*_+*q*_*p*_′/*q*+*q*′}.

**Theorem 2 .**

Let *n* > 1 be an integer such that gcd(*n*, 6) = 1. If there exist a 81-regular CDP ({3, 4}, 1, {7/8, 1/8}; 81n), and a ({3, 4}, 1, {10/11, 1/11}; 81)-GCP, then there exists a ({3, 4}, 1, {21(*n* − 1)+40/24(*n* − 1)+44, 3(*n* − 1)+4/24(*n* − 1)+44}; 81*n*)-GCP.

**Proof**

There exists a 81-regular CP ({3, 4}, 1, {7/8, 1/8}; 81*n*) and a ({3, 4}, 1, {10/11, 1/11}; 81)-GCP by Lemma 1. Apply to Theorem 2, the values of size 3 and size 4 are 21 (*n* − 1) + 40 and 3 (*n* − 1) + 4, respectively. Then, a ({3, 4}, 1, {21(*n* − 1)+40/24(*n* − 1)+44, 3(*n* − 1)+40/24(*n* − 1)+44}; 81*n*)-GCP is obtained, where *DL*(*F*)={0, ±9*n*, ±10*n*, ±18*n*, ±28*n*}.

## 4. Optimal 2-D (30 × *m*, {3,4}, 1, {1/3, 2/3}) − OOCs

In this section, the existence of optimal CDP (30*m*, {3,4}, 1, {1/3, 2/3}) is proved. At first, some input designs used in the proofs after are presented in the following examples.

**Example 2 .**

There exists an optimal CDP ({3,4}, 1, {1/3, 2/3}; *m*) for *m* = 60, 90.

**Proof**

For the case of *m*=60,  *Z*_60_≅*Z*_5_ × *Z*_12_. The base blocks of an optimal CDP({3,4},1,{1/3, 2/3}; 5 × 12) are{(0,0), (1,1), (3,3),(2,7)}, {(0,0), (0,5), (3,1),(2,10)}, {(0,0),(0,10),(1,9)}.

For the case of *m*=90,  *Z*_90_≅*Z*_5_ × *Z*_16_. The base blocks of an optimal CDP ({3,4}, 1, {1/3, 2/3}; 5 × 16) are {(0,0),(1,0),(1,4)},{(0,0),(3,2),(3,11)},{(0,0),(1,1),(3,3),(2,7)},{(0,0),(0,5),(3,13),(2,6)},{(0,0),(0,10),(1,5),(3,1)},

{(0,0),(4,14),(4,13),(3,0)}.

**Example 3 .**

There exists a 15*h*-regular CDP ({3, 4}, 1, {1/3, 2/3}; 9*h* × 15) for *h* ∈ {1,2}.

**Proof**

For the case of (*h*, *v*, *g*) = (1, 135, 15), *Z*_135_≅*Z*_5_ × *Z*_27_, the base blocks of a 15-regular CDP ({3, 4}, 1, {1/3, 2/3}; 135):

(16) $$\begin{array}{c} \left\{\left(0,0,\right),\left(0,5\right),\left(02,0\right)\right\},\\ \left\{\left(0,0,\right),\left(4,14\right),\left(2,22\right),\left(1,24\right)\right\},\\ \left\{\left(0,0,\right),\left(3,13\right),\left(1,2\right)\right\},\\ \left\{\left(0,0,\right),\left(0,25\right),\left(1,19\right),\left(3,4\right)\right\},\\ \left\{\left(0,0,\right),\left(2,7\right),\left(3,23\right),\left(2,8\right)\right\},\\ \left\{\left(0,0,\right),\left(2,17\right),\left(0.11\right)\right\},\\ \left\{\left(0,0,\right),\left(0,10\right),\left(1,11\right),\left(1,14\right)\right\},\\ \left\{\left(0,0,\right),\left(4,4\right),\left(1,7\right),\left(4,10\right)\right\},\\ \left\{\left(0,0,\right),\left(4,24\right),\left(0,23\right)\right\},\\ \left\{\left(0,0,\right),\left(2,5\right),\left(2,25\right),\left(2,13\right)\right\},\\ \left\{\left(0,0,\right),\left(1,6\right),\left(0.13\right),\left(4,5\right)\right\},\\ \left\{\left(0,0,\right),\left(3,1\right),\left(1,12\right)\right\}. \end{array}$$

For the case of (*h*, *v*, *g*) = (2, 270, 30), *Z*_270_≅*Z*_5_ × *Z*_54_, the base blocks of a 30-regular CDP ({3, 4}, 1, {1/3, 2/3}; 270):

(17) $$\begin{array}{c} \left\{\left(0,0\right),\left(0,10\right),\left(4,5\right),\left(3,31\right)\right\},\\ \left\{\left(0,0\right),\left(3,38\right),\left(0,50\right),\left(3,4\right)\right\},\\ \left\{\left(0,0\right),\left(1,1\right),\left(1,34\right)\right\},\\ \left\{\left(0,0\right),\left(3,53\right),\left(3,40\right),\left(0,42\right)\right\},\\ \left\{\left(0,0\right),\left(2,47\right),\left(4,31\right),\left(4,46\right)\right\},\\ \left\{\left(0,0\right),\left(1,6\right),\left(2,8\right)\right\},\\ \left\{\left(0,0\right),\left(0,30\right),\left(2,13\right),\left(0,52\right)\right\},\\ \left\{\left(0,0\right),\left(0,40\right),\left(2,25\right),\left(2,30\right)\right\},\\ \left\{\left(0,0\right),\left(1,11\right),\left(2,10\right)\right\},\\ \left\{\left(0,0\right),\left(0,25\right),\left(1,29\right),\left(4,32\right)\right\},\\ \left\{\left(0,0\right),\left(2,32\right),\left(4,51\right),\left(2,40\right)\right\},\\ \left\{\left(0,0\right),\left(3,13\right),\left(1,39\right)\right\},\\ \left\{\left(0,0\right),\left(1,26\right),\left(0,1\right),\left(4,22\right)\right\},\\ \left\{\left(0,0\right),\left(4,14\right),\left(3,48\right),\left(0,11\right)\right\},\\ \left\{\left(0,0\right),\left(4,19\right),\left(0,38\right)\right\},\\ \left\{\left(0,0\right),\left(1,41\right),\left(4,12\right),\left(2,35\right)\right\},\\ \left\{\left(0,0\right),\left(1,12\right),\left(2,49\right),\left(0,28\right)\right\},\\ \left\{\left(0,0\right),\left(4,24\right),\left(2,52\right)\right\},\\ \left\{\left(0,0\right),\left(4,4\right),\left(2,34\right),\left(1,24\right)\right\},\\ \left\{\left(0,0\right),\left(2,22\right),\left(2,3\right),\left(4,10\right)\right\},\\ \left\{\left(0,0\right),\left(1,31\right),\left(4,37\right)\right\},\\ \left\{\left(0,0\right),\left(1,46\right),\left(1,43\right),\left(2,5\right)\right\},\\ \left\{\left(0,0\right),\left(1,21\right),\left(0,6\right),\left(0,23\right)\right\},\\ \left\{\left(0,0\right),\left(1,7\right),\left(0,47\right)\right\}. \end{array}$$

Some results of optimal 2-D (*n* × *m*, {3, 4}, 1, {1/3, 2/3})-OOCs are obtained in [5]. The following results come from [5].

**Lemma 8 .**

If *m* ≡ 30,150(mod 180) is an integer, and *m* > 30, then there exists an optimal 2-D (1 × *m*, {3, 4}, 1, {1/3, 2/3})-OOC.

**Lemma 9 .**

If *n* is an integer such that gcd(*n*, 30)=1, *n* > 1, then there exists a 30-regular CDP ({3, 4}, 1, {1/3, 2/3}; 30*n*).

The following examples of hg-regular h-perfect CDP (*W*, 1, *Q*; *hv*) are useful to our constructions, which we state below:

**Example 4 .**

There exist:

1. *hg*-regular *h*-perfect CDP ({3,4}, 1, {1/3, 2/3}; *hm*) s for *h* ∈ {1,2}and (*m*, *g*) ∈ {(40,10), (120,30), (180,30)};
2. 30-regular CDP ({3,4}, 1, {1/3, 2/3}; *m*) s for *m* ∈ {180,360,480,540,810};
3. *g*-regular CDP ({3,4}, 1, {1/3, 2/3}; *g* × 5) s for *g* ∈ {60,90}.

**Proof**

1. For the case of (*h*, *m*, *g*) = (1, 40, 10), *Z*_40_≅*Z*_5_ × *Z*_28_, the base blocks of a 10-regular 1-perfect CDP ({3, 4}, 1, {1/3, 2/3}; 40): {(0,0),(1,1),(4,6),(4,3)}, {(0,0),(2,2),(1,3),(2,1)}, { (0, 0),(3, 3), (0,2)}.
2. For the case of (*h*, *m*, *g*) = , *Z*_40_≅*Z*_5_ × *Z*_28_, the base blocks of a 20-regular 2-perfect CDP ({3, 4}, 1, {1/3, 2/3}; 2 × 40): {(0, 0),(1, 1),(3, 3), (3,2)},{(0,0), (0,5), (1, 3),(3,10)}, {(0,0), (4, 9), (4,3), (2,10)}, {(0, 0), (1,11), (1,9), (4,6)}, {(0, 0),(1,6),(0,7)},{(0, 0), (4,14), (4,11)}.
3. For the cases of (*m*, *g*) ∈ {(120,30), (180,30)}, *Z*_*v*_≅*Z*_*s*_ × *Z*_*t*_*an*  *d* *h* ∈ {1,2}, the base blocks of hg-regular h-perfect CDP ({3, 4}, 1, {1/3, 2/3}; *m*) s are listed in Table 4
4. For the cases of *m* ∈ {180,240,360,480,540,810}, the base blocks of 30-regular CDP ({3, 4},1,{1/3, 2/3}; *m*)s are listed in Table 5:
5. For each (*g*, *m*) ∈ {(60,300), (90,450)},  *Z*_*m*_≅*Z*_*s*_ × *Z*_*t*_, a g-regular CDP ({3, 4}, 1, {1/3, 2/3}; m) is designed by listing all its codewords as Table 6:

**Lemma 10 .**

For any positive integer *i* ≥ 2, then there exists a 30-regular CDP ({3,4}, 1, {1/3, 2/3}; 30 × 3^*i*^).

**Proof**

When *Q*={1/3, 2/3}, for the cases *i*=2,3, a 30-regular CDP ({3,4}, 1, {1/3, 2/3}; 30 × 3^*i*^) comes from Examples 3 and 4, respectively.

For *i*=4, applying Construction 4, we get a 30 × 9-regular 18-perfect CDP ({3,4}, 1, {1/3, 2/3}; 30 × 3^4^), where the needed 15-regular 1-perfect CDP ({3, 4}, 1, {1/3, 2/3}; 15 × 3^2^), 30-regular 2-perfect CDP ({3, 4}, 1, {1/3, 2/3}; 30 × 3^2^) and 2-regular (18; 4; 1)-ICDM comes from Example 3 and Lemma 5. Start from this (30 × 9)-regular CDP ({3,4}, 1, {1/3, 2/3}; 30 × 3^4^), and apply Construction 2 with a 30-regular CDP ({3, 4}, 1, {1/3, 2/3}; 30 × 3^2^) to obtain a 30-regular CDP ({3, 4}, 1, {1/3, 2/3}; 30 × 3^4^). When *i* ≥ 5, start from a 30 − regular *C*  *DP*({3,4}, 1, {1/3, 2/3}; 30 × 3^*i*^) from the above with *t* ≡ *i*(mod 3) and *t*∈{2,3,4}. Apply Construction 5 with a (3^3^, 4; 1)-CDM from Lemma 4, recursively. This gives a 30-regular CDP ({3,4}, 1, {1/3, 2/3}; 30 × 3^*i*^) for *i* ≥ 5. 

**Lemma 11 .**

For any positive integer *i* ≥ 1, then there exists a 30-regular CDP ({3,4}, 1, {1/3, 2/3}; 60 × 3^*i*^).

**Proof**

When *i*={1,2}, a 30-regular CP ({3,4}, 1, {1/3, 2/3}; 60 × 3^*i*^) comes from Example 4.

When *i*=3. By Construction 4, we get a (15 × 12)-regular 15-perfect CDP ({3,4}, 1, {1/3, 2/3}; 60 × 3^3^), where the needed 15-regular 1-perfect CDP ({3,4}, 1, {1/3, 2/3}; 15 × 3^2^), 30-regular 2-perfect CDP ({3, 4}, 1, {1/3, 2/3}; 30 × 3^2^) and 2-regular (12, 4; 1)-ICDM comes from Example 4 and Lemma 5. Start from this (15 × 12)-regular 15-perfect CDP ({3,4}, 1, {1/3, 2/3}; 60 × 3^3^), and apply Construction 1 with a 30-regular CDP ({3,4}, 1, {1/3, 2/3}; 60 × 3) to obtain a 30-regular CDP ({3,4}, 1, {1/3, 2/3}; 60 × 3^3^).

When *i* ≥ 4, the parameter *i* can be written as *i*=3*s*+*t* where *s* ≥ 1 and *t* = 1, 2, 3. Start from a 30-regular CDP ({3,4}, 1, {1/3, 2/3}; 60 × 3^*t*^) from above. Apply Construction 4*g*=30, *m*=3^3*s*^, and *v*=60 × 3^*t*^ to obtain a 30-regular CDP ({3,4}, 1, {1/3, 2/3}; 60 × 3^*t*^) for *i* ≥ 4, where the needed 30-regular CDP ({3,4}, 1, {1/3, 2/3}; 30 × 3^*s*^) and (3^3*s*^, 4; 1)-CDM exist by Lemmas 4 and 10.

**Lemma 12 .**

If *m* is a positive integer such that gcd(*m*, 30)=1, then there exists a 30-regular CDP ({3,4}, 1, {1/3, 2/3}; *gu* × 3^*i*^) for *g* = {60, 90} and *i* ≥ 1.

**Proof**

For *i* ≥ 1, there exists a 30-regular CDP ({3,4}, 1, {1/3, 2/3}; *g* × 3^*i*^) for *g* = {60, 90} by Lemmas 10 and 11. Start from a 30-regular CDP ({3,4}, 1, {1/3, 2/3}; 30 × *m*) for gcd(*m*, 30)=1 from Lemma 9. Then, apply Construction 2 with a (*u*, 4; 1)-CDM from Lemma 4 to obtain a 30-regular CDP ({3,4}, 1, {1/3, 2/3}; *gu* × 3^*i*^).

**Lemma 13 .**

For any positive integer *i* ≥ 2, then there exists a 30-regular CDP ({3,4}, 1, {1/3, 2/3}; 30 × 2^*i*^).

**Proof**

For *i*=2,3,4, a 30-regular CDP ({3,4}, 1, {1/3, 2/3}; 30 × 2^*i*^) exists by Example 4. Next, we consider the case of *i* ≥ 5. Begin with a 30-regular 1-perfect CDP ({3,4}, 1, {1/3, 2/3}; 30 × 2^2^) by Example 4. Take a 2-perfect (2^*i*−2^, 4; 1)-ICDM from Lemma 5. Then, apply Construction 4 with *g*=30, *m*=2^*i*−2^, *h*=2, and *v*=30 × 2^2^ to obtain a (30 × 2^*i*−2^)-regular CDP ({3, 4}, 1, {1/3, 2/3}; 30 × 2^*i*^). Combining with a 30-regular CDP ({3, 4}, 1, {1/3, 2/3}; 30 × 2^3^) and a 30-regular CDP({3, 4}, 1, {1/3, 2/3}; 30 × 2^4^) from above, we apply Construction 1 inductively on *i* to get a 30-regular CDP({3, 4}, 1, {1/3, 2/3}; 30 × 2^*i*^) for any integer *i* ≥ 5.

**Lemma 14 .**

For any positive integer *i* ≥ 1, then there exists a 30-regular CDP ({3,4}, 1, {1/3, 2/3}; 90 × 2^*i*^).

**Proof**

For *i*=1,2, a 30-regular CDP ({3,4}, 1, {1/3, 2/3}; 90 × 2^*i*^) exists by Example 4. Next, we consider the case of *i*=3. Begin with a 10-regular 1-perfect CDP ({3,4}, 1, {1/3, 2/3}; 40) and a 20-regular 2-perfect CDP ({3, 4}, 1, {1/3, 2/3}; 80) by Example 4. Take a 2-perfect (18, 4; 1)-ICDM from Lemma 5. Then, apply 1 with *g*=30, *m*=2^*i*−2^, *h*=2, and *v*=40 to obtain a (90 × 2)-regular CDP ({3,4}, 1, {1/3, 2/3}; 90 × 2^3^). Combining with a 30-regular CDP ({3,4}, 1, {1/3, 2/3}; 90 × 2) from above, we apply 1 to get a 30-regular CDP ({3,4}, 1, {1/3, 2/3}; 90 × 2^3^).

Now, we deal with the case of *i* ≥ 4. Start from a 30-regular 1-perfect CDP ({3,4}, 1, {1/3, 2/3}; 30 × 6) and a 60-regular 2-perfect CDP ({3,4}, 1, {1/3, 2/3}; 60 × 6) by Example 4. Take a 2-regular (2^*i*−1^, 4; 1)-ICDM from Lemma 5. Then, we apply 4*with* *g*=30, *m*=2^*i*−2^, *h*=2, and *v*=30 × 6 to obtain a (30 × 2^*i*−1^)-regular CDP ({3,4}, 1, {1/3, 2/3}; 90 × 2^*i*^). Combining with Lemma 13, there exists a 30-regular CDP ({3,4}, 1, {1/3, 2/3}; 30 × 2^*i*−1^). We apply 1 to get a 30-regular CDP ({3,4}, 1, {1/3, 2/3}; 90 × 2^*i*^).

**Lemma 15 .**

For positive integer *i*, *j* ≥ 2, then there exists a 30-regular CDP ({3,4}, 1, {1/3, 2/3}; 30 × 2^*i*^3^*j*^).

**Proof**

For *i*=2 and *j*=2, begin with a 15-regular CDP ({3,4}, 1, {1/3, 2/3}; 9 × 15) and a 30-regular CDP ({3,4}, 1, {1/3, 2/3}; 9 × 30) respectively, which exist by Example 3. Take a 2-regular (2^*i* + 1^, 4; 1)-ICDM from Lemma 5. Next, apply 4 with *g* = 15, *m* = 2*i*+1, *h* = 2 and *v*=9 × 15 to obtain a (30 × 2^*i*^)-regular CDP ({3,4}, 1, {1/3, 2/3}; 30 × 2^*i*^3^2^).

There exists a 30-regular CDP ({3,4}, 1, {1/3, 2/3}; 30 × 2^*i*^) by Lemma 13. We apply 1 to obtain a 30-regular CDP ({3,4}, 1, {1/3, 2/3}; 30 × 2^*i*^3^2^).

For the case of *i* ≥ 2 and *j* ≥ 3. Begin with a 30-regular CDP ({3,4}, 1, {1/3, 2/3}; 30 × 2^*i*^) and a (3^*j*^, 4; 1)-CDM, and a 30-regular CDP ({3,4}, 1, {1/3, 2/3}; 30 × 3^*i*^), which exist by Lemma 13, Lemma 4 and Lemma 10, respectively. Then, apply 3 with *g* = 30, *m* =  3^*j*^ and *v*=30 × 2^*i*^ to obtain a 30-regular CDP ({3,4}, 1, {1/3, 2/3}; 30 × 2^*i*^3^*j*^).

**Lemma 16 .**

If *g*={60,90}and *k* ≥ 1, then there exists a g-regular CDP ({3,4}, 1, {1/3, 2/3}; *g* × 5^*k*^).

**Proof**

For *g* = {60, 90}, a g-regular CDP ({3,4}, 1, {1/3, 2/3}; *g* × 5) exists by Example 4. For the case *of* *k* ≥ 1. Begin with a g-regular CDP ({3,4}, 1, {1/3, 2/3}; *g* × 5), then apply 1 inductively with a (5; 4; 1)-CDM from Lemma 3 to obtain a g-regular CDP ({3,4}, 1, {1/3, 2/3}; *g* × 5^*k*^).

**Lemma 17 .**

For any positive integer *i* ≥ 2, *k* ≥ 1, then there exists a 30-regular CDP ({3,4}, 1, {1/3, 2/3}; 30 × 2^*i*^5^*k*^) .

**Proof**

For *i* ≥ 2 and *k* ≥ 1, begin with a 30-regular CDP (({3,4}, 1, {1/3, 2/3}; 30 × 2^*i*^) and a (5^*k*^; 4; 1)-CDM, respectively, which exist by Example 4.9 and Lemma 4 and Lemma 13. Next, apply 2 to obtain a (30 × 5^*k*^)-regular CDP ({3,4}, 1, {1/3, 2/3}; 30 × 2^*i*^5^*k*^). There exists a 30-regular CDP ({3,4}, 1, {1/3, 2/3}; 30 × 5^*k*^) by the result in [21]. We apply 1 to obtain a 30-regular CP ({3,4}, 1, {1/3, 2/3}; 30 × 2^*i*^5^*k*^).

**Lemma 18 .**

For any positive integer *j* ≥ 2, *k* ≥ 1, then there exists a 30-regular CDP({3,4}, 1, {1/3, 2/3}; 30 × 3^*j*^5^*k*^).

**Proof**

For *j* ≥ 2 and *k* ≥ 1, begin with a 30-regular CDP ({3,4}, 1, {1/3, 2/3}; 30 × 3^*j*^) and a (5^*k*^; 4; 1)-CDM, respectively, which exist by Lemmas 4 and 10. Next, apply 2 to obtain a (30 × 5^*k*^)-regular CDP ({3,4}, 1, {1/3, 2/3}; 30 × 3^*j*^5^*k*^). There exists a 30-regular CDP ({3,4}, 1, {1/3, 2/3}; 30 × 5^*k*^) by Lemma 17 We apply 1 to obtain a 30-regular CDP ({3,4}, 1, {1/3, 2/3}; 30 × 3^*j*^5^*k*^).

**Lemma 19 .**

For any positive integer *u* > 1, then there exists an optimal CDP ({3,4}, 1, {1/3, 2/3}; 30*u*).

**Proof**

Suppose *u*=2^*i*^3^*j*^5^*k*^*u*′*such* *that* gcd(*u*′, 30)=1. For *Q* = {1/3, 2/3}, we have the following two cases.

**Step 1 .**

when *u*′=1, , then 30*u*=30 × 2^*i*^3^*j*^5^*k*^*u*′.

**Step 2 .**

:If *k* = 0, then 30 *u*=30 × 2^*i*^3^*j*^. If *i*=0, then *j* ≥ 1. When *j*=1, there is an optimal CDP ({3,4}, 1, {1/3, 2/3}; 90) by Example 2. When *j* ≥ 2, there is a 30-regular CDP ({3,4}, 1, {1/3, 2/3}; 30 × 3^*j*^) by Lemma 10. If *i*=1, then *j* ≥ 0. When *j* = 0, there is an optimal CDP ({3, 4}, 1, {1/3, 2/3}; 60) by Example 2. When *j* ≥ 1, there is a 30-regular CDP ({3,4}, 1, {1/3, 2/3}; 60 × 3^*j*^) by Lemma 11. If *i* ≥ 2, then *j* ≥ 0, there exists a 30-regular CDP ({3,4}, 1, {1/3, 2/3}; 30 × 2^*i*^3^*j*^) Lemmas 13–15.

**Step 3 .**

If *k* ≥ 1, then we have three subcases.

- If *i*=0, then *j* ≥ 0. When *j*=0, there is an 30-regular CDP ({3,4}, 1, {1/3, 2/3}; 30 × 5^*k*^). When *j* ≥ 0, there is a 90-regular CDP ({3,4}, 1, {1/3, 2/3}; 90 × 5^*k*^) by Lemma 16. Take an optimal CDP({3,4}, 1, {1/3, 2/3}; 90) from Example 2, then apply 1 to get an optimal CDP({3,4}, 1, {1/3, 2/3}; 90 × 5^*k*^). When *j* ≥ 2, there exists a 30-regular CDP ({3,4}, 1, {1/3, 2/3}; 30 × 3^*j*^5^*k*^) by Lemma 18.
- If *j*=0, then *i* ≥ 1. When *i*=1, there is a 60-regular CDP ({3,4}, 1, {1/3, 2/3}; 60 × 5^*k*^) by Lemma 16. Take an optimal CDP ({3,4}, 1, {1/3, 2/3}; 60) from Example 2, then apply 1 to get an optimal CDP ({3,4}, 1, {1/3, 2/3}; 60 × 5^*k*^). When *i* ≥ 2, there exists a 30-regular CDP ({3,4}, 1, {1/3, 2/3}; 30 × 2^*i*^5^*k*^) by Lemma 17.
- If *i* ≥ 1 and*j* ≥ 1, start from a 30-regular CDP ({3,4}, 1, {1/3, 2/3}; 30 × 2^*i*^3^*j*^) which exists by the Step 2. Then, apply 1 to get a (30 × 5^*k*^)-regular CDP ({3,4}, 1, {1/3, 2/3}; 30 × 2^*i*^3^*j*^5^*k*^), where the needed a (5^*k*^, 4; 1)-CDM comes from Lemma 4. Furthermore, take a 30-regular CDP({3,4}, 1, {1/3, 2/3}; 30 × 5^*k*^) from [21], apply 1 to get a 30-regular CDP ({3,4}, 1, {1/3, 2/3}; 30 × 2^*i*^3^*j*^5^*k*^).

**Step 4 .**

when *u*′>1, then 30*u*=2^*i*^3^*j*^5^*k*^*u*′.

**Step 5 .**

If *k*=0, then there have three subcases.

- If *i*=0, then *j* ≥ 0. When *j*=0, there is a 30-regular CDP ({3,4}, 1, {1/3, 2/3}; 30*u*) by Lemma 9. When *j* ≥ 1, there is a 90-regular CDP ({3,4}, 1, {1/3, 2/3}; 90*u*′) from Lemma 7, then we apply 3 to get an optimal CDP ({3,4}, 1, {1/3, 2/3}; 90*u*′), where the needed optimal CDP ({3,4}, 1, {1/3, 2/3}; 90) comes from Example 2. When *j* ≥ 2, there is a 30-regular CDP ({3,4}, 1, {1/3, 2/3}; 30 × 3^*j*^*u*′) by Lemma 10.
- If *i*=1, then *j* ≥ 0. When *j*=0, there is a 60-regular CDP ({3,4}, 1, {1/3, 2/3}; 60*u*′), and an optimal CDP ({3,4}, 1, {1/3, 2/3}; 60), which come from Lemma 7 and Example 2, respectively. Then, we apply 2 to get an optimal CDP ({3,4}, 1, {1/3, 2/3}; 60*u*′). When *j* ≥ 1, there is a 30-regular CDP ({3,4}, 1, {1/3, 2/3}; 60 × 3^*j*^) by Lemma 11.
- If *i* ≥ 2, then *j* ≥ 0. Start from a 30-regular CDP ({3,4}, 1, {1/3, 2/3}; 30 × 2^*i*^3^*j*^), which exists by Lemmas 13–15. Take a 30-regular CDP ({3,4}, 1, {1/3, 2/3}; 30 × 2^*i*^3^*j*^) from Lemma 15. Then, we apply 2 with a (*u*′, 4; 1)-CDM from Lemma 4, to get a 30-regular ({3,4}, 1, {1/3, 2/3}; 30 × 2^*i*^3^*j*^*u* ′). It is a 30-regular CDP ({3,4}, 1, {1/3, 2/3}; 30*u*). According to Lemma 2, the resulting 30-regular CDP ({3,4}, 1, {1/3, 2/3}; 30*u*) from above is optimal.

**Step 6 .**

For *k* ≥ 1. There exists a 30-regular CDP ({3,4}, 1, {1/3, 2/3}; 30 × 2^*i*^3^*j*^*u* ′) from the Step 5. Then, we apply 2 with a (5k, 4; 1)-CDM from Lemma 4 obtain a (30 × 5^*k*^)-regular CDP ({3,4}, 1, {1/3, 2/3}; 30 × 2^*i*^3^*j*^5^*k*^*u* ′). We can get a 30-regular CDP ({3,4}, 1, {1/3, 2/3}; 30 × 2^*i*^3^*j*^*u*′)with 1. Similar to the abovementioned statements, the needed 30-regular CDP ({3,4}, 1, {1/3, 2/3}; 30 × 5^*k*^) comes from [1].

**Step 7 .**

By Lemma 2, the resulting 30-regular CDPs from the above are all optimal. Combined with the above proofs, we can obtain a new family of optimal 2-D (*n* × *m*, {3,4}, 1, {1/3, 2/3})-OOCs.

## 5. Conclusion

Two-dimensional (2-D) multiple-weight optical orthogonal codes are of great importance to enable optical communication at lower chip rate to overcome the drawbacks of nonlinear effects in large spreading sequences of one-dimensional codes. In this paper, we have focused our attention on the investigations of 2-D OOCs by combinatorial methods. Specifically, an improved class of skew starters with multiple weights is given and the existence results of optimal multiple-weight optical orthogonal codes are updated. Through incomplete difference matrix, h-perfect cyclic packing and skew starter, we establish a family of optimal multiple-weight optical orthogonal codes that can support quality service for a distinct service with given multiple factors. This work can help to meet multiple quality services for the demands of different quality services for different services and distinct subscribers so as to optimize the utilization of optical network effectively.

On the other hand, we mainly study the structures of optimal (*v*; *W*,1,*Q*)-OOCs with *W* = {3,4}. As we know, the results of (*v*; *W*,1,*Q*)-OOCs are little, when |*W*| ≥ 3. This shows that the following problems should studying in the further research studies, such as *W* = {3,4,6}, {3,5,7}, {4,5,6}, and {3,4,5,6}.

## Figures and Tables

**Table 1:** Values of differences of 60*n*.

*D*_*s*_	The values of *s*
∪_*i*=1_^*t*^{±(*u*_*i*_+*v*_*i*_)}	{3, 4, 7, 8,13, 15, 23, 25, 30, 38, 47}
∪_*i*=1_^*t*^{±(*u*_*i*_ − *v*_*i*_)}	{0, 2, 9, 10, 11, 18, 39, 41, 43}
∪_*i*=1_^*t*^{±(−2*u*_*i*_ − 2*v*_*i*_)}	{6,36}
∪_*i*=1_^*t*^{±2*u*_*i*_}	{5, 14, 16, 26}
∪_*i*=1_^*t*^{±2*v*_*i*_}	{32, 33, 40}
∪_*i*=1_^*t*^{±(*u*_*i*_, *v*_*i*_)}	{1}
∪_*i*=1_^*t*^{±2(*u*_*i*_+*v*_*i*_)}	{12}
∪_*i*=1_^*t*^{±(−*u*_*i*_, −*v*_*i*_)}	{29}

**Table 2:** Values of differences of 90*n*.

*D*_*s*_	The values of *s*
∪_*i*=1_^*t*^{±(*u*_*i*_+*v*_*i*_)}	{3, 4, 6, 7, 8, 9, 10, 15, 16, 21, 24, 31, 33, 39, 45}
∪_*i*=1_^*t*^{±(*u*_*i*_ − *v*_*i*_)}	{0, 2, 11, 12, 13, 14, 18, 26, 27, 28, 29, 30, 32, 38}
∪_*i*=1_^*t*^{(−2*u*_*i*_, −2*v*_*i*_)}	{20, 25}
∪_*i*=1_^*t*^{±2*u*_*i*_}	{5, 19, 23, 36, 37, 42, 43}
∪_*i*=1_^*t*^{(*u*_*i*_, *v*_*i*_)}	{35, 41, 34, 22,17}
∪_*i*=1_^*t*^{±2*v*_*i*_}	{1}
∪_*i*=1_^*t*^{±2(*u*_*i*_+*v*_*i*_)}	{40}
∪_*i*=1_^*t*^{(−*u*_*i*_, −*v*_*i*_)}	{44}

**Table 3:** ({3, 4}, 1, *Q*; *g*)-GCPs.

*g*	*Q*	{*a*} or {*a*, *b*}
45	{4/5, 1/5}	{5}
81	{10/11, 1/11}	{9}
48	{3/4, 1/4}	{3,14}
48	{1/3, 2/3}	{3,14}
54	{1/2, 1/2}	{3,16}
60	{5/6, 1/6}	{11,24}
72	{7/8, 1/8}	{11,28}
90	{2/7, 5/7}	{15,18}

**Table 4:** Some *hg*-regular *h*-perfect CDP ({3,4}, 1, {1/3, 2/3}; *hm*) s of Example 4.

*h*	(*m*, *g*, *s*, *t*)	Codewords
1	(120,30,5,24)	{(0,0),(1,1), (1,3), (4, 6)}, {(0,0),(3,18), (2,13),(3,19)}, {(0, 0),(4,9),(0,7)}, {(0,0),(4,14),(1,21),(2,23)}, {(0,0),(1,11),(4,10),(4,1)}, {(0,0),(3,13),(3,10)}, {(0,0),(0,6),(0,11),(2,9)}, {(0,0),(2,2),(1,7),(1,17)}, {(0,0),(2,17),(4,11)}.
	(180,30,5,36)	{(0,0),(1,26),(4,34), (0,13)}, {(0,0),(2,7), (1,35),(3,16)}, {(0,0),(4,29),(2,15)}, {(0,0),(3,3),(0,19),(1,14)}, {(0,0),(2,22),(2,11),(2,26)}, {(0,0),(3,17),(3,1)}, {(0, 0),(0,10),(4,14),(2,5)}, {(0,0),(1,16),(2,27),(0,29)}, {(0,0),(3,32),(4,17}, {(0,0),(3,23),(4,7),(0,8)}, {(0,0),(0,35),(4,8),(1,4)}, {(0,0),(0,14),(4,33)}, {(0,0),(2,1),(4,3),(2,10)}, {(0,0),(3,13),(1,10),(4,2)}, {(0,0),(0,34), (0,3)}

2	(120,60,5,48)	{(0,0),(2,27),(2,18),(4,25)}, {(0,0),(2,26),(4,43),(2,33)}, {(0,0),(2,22),(0,29)}, {(0,0),(1,1), (0,35),(1,22)}, {(0,0),(1,26),(1,27), (3,29)}, {(0,0),(2,42),(4,33)}, {(0,0),(1,46),(2,9),(3,27)}, {(0,0),(4,9),(4,11),(0,6)}, {(0,0),(3,23),(3,34)}, {(0,0),(4,39),(3,5),(3,10)}, {(0,0),(1,21),(4,6),(0,31)}, {(0,0),(4,1),(4,35)}, {(0,0),(0,45),(4,38),(4,15)}, {(0,0),(0,10),(1,41),(2,47)}, {(0,0),(4,29),(2,23)}, {(0,0),(3,47),(1,2),(1,17)}, {(0,0),(3,13),(3,43),(0,26)}, {(0,0),(1,3),(3,37)}
		{(0,0), (1,11),(1,9),(4,13)}, {(0,0),(0,55),(2,62),(0,41)}, {(0,0),(2,17),(2,67)}, {(0,0),(0,15),(3,59),(1,50)}, {(0,0),(1,26),(2,41),(2,51)}, {(0,0),(4,29),(2,46)}, {(0,0),(1,56),(2,5),(3,7)}, {(0,0),(2,32),(4,69),(0,29)}, {(0,0),(3,68),(4,43)}, {(0,0),(4,4),(0,3), (4,17)}, {(0,0),(4,44),(0,51), (4,28)}, {(0,0),(0,25),(2,16)}, {(0,0),(4,34),(0,65),(2,1)}, {(0,0),(3,43),(2,10),(3,11)}, {(0,0),(1,46),(0,49)}
	(180,60,5,72)	{(0,0),(2,27),(4,7), (0,46)}, {(0,0),(2,38),(2,58),(0,39)}, {(0,0),(1,4),(4,50)}, {(0,0),(3,13), (4,8),(4,53)}, {(0,0),(3,8),(1,41),(1,45)}, {(0,0),(0,5),(3,52)}, {(0,0), (3,16),(0,61),(2,11)}, {(0,0), (4,19), (0,8), (0,9)}, {(0,0),(3,28),(4,38)}, {(0,0),(2,57),(4,59), (1,37)}, {(0,0),(1,14), (2,31),(0,34)}, {(0,0),(4,64),(4,45)}, {(0,0),(1,16), (1,51),(4,2)}, {(0,0), (1,57), (4,23),(3,32)}, {(0,0),(2,15),(2,43)}.

**Table 5:** The base blocks of 30-regular CDP ({3, 4}, 1, {1/3, 2/3}; *m*)s of Example 4.

(*g*, *m*, *s*, *t*)	Codewords
(30,180,5,36)	{(0,0),(2,1), (4,3), (2,10)}, {(0,0),(3,23), (4,7),(0,8) }, {(0,0), (0,34),(0,3)}, {(0,0),(3,13),(1,10),(4,2)}, {(0,0), (0,35), (4,8),(1,4)}, {(0, 0),(0,14),(4,33)}, {(0,0),(3,3), (0,19),(1,14)}, {(0,0), (2,22), (2,11),(2,26)}, {(0,0), (3,17), (3,1)}, {(0,0),(0,10),(4,14),(2,5)}, {(0,0), (1,16),(2,27), (0,29) }, {(0, 0),(3,32),(4,17)}, {(0,0), (1,26),(4,34),(0,13)}, {(0,0),(2,7),(1,35),(3,16)}, {(0,0),(4,29), (2,15)}

(30,360,5,72)	{(0,0),(3,54), (3,52), (1,65)}, {(0,0), (2,58),(2,31), (1,28)}, {(0,0),(2,3),(0,71)}, {(0,0),(2,47),(3,56), (4,21)}, {(0,0),(2,21),(1, 55),(2,29)}, {(0,0),(0,25),(2,30)}, {(0,0),(1,16),(1,27), (2,33)}, {(0,0),(2,17),(4,1),(4,11)}, {(0,0), (0,40),(2,23)}, {(0,0),(2,22),(4,13),(3,65) }, {(0,0),(3,18),(4,47),(3,2) }, {(0,0), (3,1),(0,38)}, {(0,0),(3,53),(4,25), (1,15) }, {(0,0),(2,42),(4,10),(3,47) }, {(0,0),(1,7), (4,6)}, {(0,0),(0,31),(1,52), (1,57)}, {(0,0), (2,10), (1,18),(3,20)}, {(0,0), (2,11), (2,39)}, {(0,0),(1,39),(0,26), (0,69)}, {(0,0), (3,19), (3, 40),(4,41)}, {(0,0), (1,14),(1,8)}, {(0,0),(3,8),(4,31), (2,69)}, {(0,0),(4,19),(4,38), (1,33)}, {(0,0),(3,31), (0,4)}, {(0,0), (2,35), (0,58),(1,40)}, {(0,0), (4,14), (0,63), (2,6)}, {(0,0),(0,15), (0,52)}, {(0,0), (1,4),(0,7),(1,63)}, {(0,0),(2,28),(0, 49),(1,68)}, {(0,0),(0,39),(0,17)}, {(0,0),(1,2), (3,15), (3,45)}, {(0,0), (3,4),(3,22),(1,50)}, {(0,0),(3,63),(2, 65)}

(30,480,5,96)	{(0,0), (4,34),(0,83), (4,61)}, {(0,0),(4,23), (2,25), (0,78)}, {(0,0),(2,46),(4,1)}, {(0,0),(2,27),(0,73),(1,42)}, {(0,0),(1,21), (2,30), (2,88)}, {(0,0),(3,83), (3,36)}, {(0,0),(3,72),(0,37),(1,63)}, {(0,0),(4,39),(4,73), (1,83)}, {(0, 0),(3,68), (4,8)}, {(0,0),(3,33),(1,75),(0,67)}, {(0,0),(2,37),(4,3), (1,18)}, {(0,0),(1,6), (4,46)}, {(0,0),(1,86),(4,57),(2,68)}, {(0,0),(4,44),(3,93),(2,66)}, {(0,0),(4,22),(0,36)}, {(0,0),(4,14),(1,90),(1,84)}, {(0,0),(2,52),(3,77),(2,53)}, {(0,0),(1,71),(2,18)}, {(0,0),(4,19),(1,30),(1,4)}, {(0,0),(2,57),(2,82), (2,36)}, {(0,0),(0,10),(2,87)}, {(0,0),(0,20),(1,66), (2,55)}, {(0,0),(3,88),(2,86), (2,20)}, {(0,0),(1,1), (0,5)}, {(0,0),(1,76), (2,31),(3,29)}, {(0,0),(3,27),(0,74),(3,51)}, {(0,0),(2,26),(2,91)}, {(0,0),(4,79),(4,93),(4,81)}, {(0,0),(2,2),(4,86), (1,7)}, {(0,0),(4,24), (2,41)}, {(0,0),(0,40),(0,7),(0,92)}, {(0,0),(0,39),(2,14),(4,26)}, {(0,0),(3,7),(0,28)}, {(0,0),(0,15),(2,22),(1,60)}, {(0,0),(3,58),(1,61),(2,5)}, {(0,0),(3,38),(0,17)}, {(0,0),(0,35),(0,54),(4,42)}, {(0,0),(3,13),(0,53),(3,54)}, {(0,0),(4,37),(1,38)}, {(0,0), (4,9),(2,72), (3,4)}, {(0,0),(3,18),(4,59),(4,62)}, {(0,0),(0,9),(4,76)}

(30,540,5,108)	{(0,0),(1,13),(4,8), (2,43)}, {(0,0),(1,83),(1,17),(1,57)}, {(0,0),(2,102),(0,19)}, {(0,0),(3,50),(1,58),(1,63)}, {(0,0),(3,33),(3,83),(4,10)}, {(0,0),(4,33),(3,46)}, {(0,0),(2,16),(4,28),(2,55)}, {(0,0),(2,27),(0,3), (1,29)}, {(0,0),(4,104),(3,34)}, {(0,0),(0,15),(1,96),(1,84)}, {(0,0),(1,8),(0,34), (3,76)}, {(0,0), (3,70),(0,33)}, {(0,0),(4,59),(1,2),(4,30)}, {(0,0), (1,6),(4,9),(1,37)}, {(0,0),(4,99), (1,22)}, {(0,0),(2,77), (2,61),(4,83)}, {(0,0),(3,32),(4,60),(4,47)}, {(0,0),(0,2), (2,44)}, {(0,0),(2,52),(2,30),(0,53)}, {(0,0),(4,49), (2,34),(4,22)}, {(0,0),(1,66),(0,63)}, {(0,0),(0,62), (1,45),(4,52)}, {(0,0),(3,100),(0,84),(0,98)}, {(0,0),(2,19), (4,107)}, {(0,0),(2,11),(3,52),(3,51)}, {(0,0),(2,21),(1,50), (3,41)}, {(0,0),(2, 64),(2,53)}, {(0,0),(3,63),(0,102),(1,87)}, {(0,0),(4,34),(0,99),(0,23)}, {(0,0),(2,17),(1,33)}, {(0,0),(0,37), (4,85),(3,104)}, {(0,0),(1,21),(2,97),(0,28)}, {(0,0),(4,81),(3,26)}, {(0,0),(4,89),(0,100),(0,52)}, {(0,0),(4,14),(3,88),(1,103)}, {(0,0),(2,7), (0,101)}, {(0,0),(4,1),(2,63),(1,24)}, {(0,0),(3,10),(4,56),(1,7)}, {(0,0),(4,66), (3,61)}, {(0,0),(0,70),(3,5),(3,22)}, {(0,0),(2,29),(2,49),(0,87)}, {(0,0),(0,57),(4,77)}, {(0,0),(4,4), (3,68),(0,47)}, {(0,0),(0,35),(1,102),(4,92)}, {(0,0),(2,2),(3,14)}, {(0,0),(2,79), (2,35),(0,83)}, {(0,0),(0,30),(4,61),(1,62)}, {(0,0),(4,94),(0,59)}

(30,810,5,162)	{(0,0),(4,47), (0,98),(2,149) }, {(0,0),(1,16),(3,103), (1,123)}, {(0,0),(0,90),(0,38)}, {(0,0),(1,49),(1,154),(3,105)}, {(0,0),(1,36),(4,38),(4,71)}, {(0,0),(3,126),(0,2)}, {(0,0),(4,64),(4,28), (2,111)}, {(0,0),(2,105),(3,109),(2,154)}, {(0,0), (4,44),(2,66)}, {(0,0),(4,59),(4,105),(4,91) }, {(0,0),(0,100),(0,24),(3,15)}, {(0,0),(0,95),(1,59)}, {(0,0),(1,79), (0,153),(1,122)}, {(0,0), (1,114),(1,17),(0,134)}, {(0,0),(3,34),(0,84)}, {(0,0),(4,32),(3,37),(3,85)}, {(0,0),(4,139),(1,159),(3,79)}, {(0,0),(2,107),(2,8)}, {(0,0),(1,44),(3,40), (0,112)}, {(0,0),(1,84),(0,118),(4,127)}, {(0,0),(3,56),(1,68)}, {(0,0),(2,37),(3,14),(1,158)}, {(0,0),(2,67),(1,104), (3,32) }, {(0,0),(3,28),(2,94) }, {(0,0),(3,59),(2,29),(3,130) }, {(0,0),(1,86),(3,151),(1,7)}, {(0,0),(4,24),(3,131)}, {(0,0),(0,150),(2,30),(0,147)}, {(0,0),(3,11),(1,32),(4,161)}, {(0,0),(0,30),(2,114)}, {(0,0),(3,29),(4,13),(0,34)}, {(0,0),(0,1),(3,137),(3,115)}, {(0,0),(2,157),(0,89)}, {(0,0),(1,76),(4,60),(2,61)}, {(0,0),(3,91),(1,72),(1,133)}, {(0,0),(4,114),(0,93)}, {(0,0),(3,53),(4,95),(3,45)}, {(0,0),(0,13),(4,101), (2,159)}, {(0,0),(2,80),(3,149)}, {(0,0),(2,152),(2,96),(3,127)}, {(0,0),(1,99),(4,140),(0,17)}, {(0,0),(0,75),(4,142)}, {(0,0),(3,73),(1,9),(4,55)}, {(0,0),(4,65),(4,85),(3,67)}, {(0,0),(1,89),(3,147)}, {(0,0),(3,86),(2,143),(0,42)}, {(0,0),(0,123),(0,41),(0,94)}, {(0,0),(1,56),(1,25)}, {(0,0),(2,132),(2,73),(4,136)}, {(0,0),(1,62),(2,6),(4,98)}, {(0,0),(4,122),(4,75)}, {(0,0),(4,99),(3,9),(1,47)}, {(0,0),(3,33),(3,26),(1,5)}, {(0,0),(2,12),(2,97)}, {(0,0),(4,49),(3,63),(4,109)}, {(0,0),(2,7),(4,62),(1,132)}, {(0,0),(0,88),(4,50)}, {(0,0),(3,23),(2,100),(0,66)}, {(0,0),(1,119),(0,104),(1,8)}, {(0,0),(1,161), (0,6)}, {(0,0),(0,10),(4,143),(0,137)}, {(0,0),(4,104),(1,28),(1,73)}, {(0,0),(3,113),(2,123)}, {(0,0),(2,112),(1,34),(4,41)}, {(0,0),(0,5),(1,116),(2,74)}, {(0,0),(3,123),(2,156)}

**Table 6:** Some 30-regular CDP ({3, 4}, 1, {1/3, 2/3}; *m*) s of Example 4.

(*g*, *m*, *s*, *t*)	Codewords
(60,300,5,60)	{(0,0), (2,14),(1,23),(0,26)}, {(0,0), (1,9), (3,67),(1,28)}, {(0,0),(2,7), (1,43)}, {(0,0), (0,12),(2,3), (0,54)}, {(0,0), (1,41),(1,34), (1,3)}, {(0,0), (3,27),(2,23)}, {(0,0), (2,34),(0,53),(0,66)}, {(0,0),(2,62),(1,38),(2,44)}, {(0,0), (1,33),(1, 62)}, {(0,0), (0,28), (0,32),(2,74)}, {(0,0), (0,16),(0,52),(3,74)}, {(0,0),(0,24),(3,57)}, {(0,0), (2,2),(1,31), (3,53)}, {(0,0), (1,29), (1, 2),(0,3)}, {(0,0),(0,61),(0,69)}, {(0,0), (2,26),(0,34), (3,62)}, {(0,0), (2,18),(1,61), (1,44)}, {(0,0),(3,19), (1,73)}, {(0,0), (3,11),(3,12), (2,28)}, {(0,0), (2,6),(1,14), (1,12)}, {(0,0), (3,23), (2,4)}

(90,450,9,50)	{(0,0), (2,2), (5, 3),(2,34)}, {(0,0), (1,32), (0,34), (7,8)}, {(0,0), (1,37), (1,4)}, {(0,0), (1,28),(5,7),(3,49)}, {(0, 0), (8,8),(5,32), (5,26)}, {(0,0),(3,16),(2,19)}, {(0,0), (4,22), (7,3),(7,39)}, {(0,0), (7,7), (0,13), (8,34)}, {(0,0), (1,41), (5,19)}, {(0,0), (5,31), (1,39), (1,43)}, {(0,0), (7,36), (5, 29), (6, 48)}, {(0,0), (2,38),(8,42)}, {(0,0), (5,44),(5,33),(5, 42)}, {(0,0),(4,13),(0,27), (4,39)}, {(0,0), (7,38),(6,16)}, {(0,0), (6,27),(3,41),(4,9)}, {(0,0),(8,33),(6,39), (6,47)}, {(0, 0), (0,31), (1,7)}, {(0,0), (8,44),(6,41),(0,47)}, {(0, 0), (3,39), (7,33), (7,26)}, {(0, 0),(8,38), (0,1)}, {(0,0), (0,22),(3, 43),(7,9)}, {(0,0),(1,14),(5,18),(3,37)}, {(0, 0), (5,9), (1,36)}, {(0,0), (7,34), (3,7),(1,11)}, {(0,0), (7,1),(2,27), (7,13)}, {(0,0),(6,6), (4,34)}, {(0,0), (1,1),(5,4),(2,32)}, {(0,0),(7,11),(4,7),(1, 24)}, {(0,0),(2,28), (7,17)}, {(0,0), (8,16),(2,4),(5,2)}, {(0,0),(8,16), (2,4),(5,2)}, {(0, 0),(5,17),(8,29)}, {(0,0), (7,2),(8, 48),(5,1)}, {(0,0),(8,6),(0,29), (3,8)}, {(0,0), (2,29),(8,1)}

## Data Availability

The data used to support the findings of this study are included within the article.
